The article "Ontology-Based Relational Product Recommendation System" was published in 2022. Journal: Comput Math Methods Med.

# Ontology-Based Relational Product Recommendation System

**DOI:** 10.1155/2022/1591044

**Published:** 2022-09-19

**Authors:** Aisha Alsobhi, Ngiste Amare

**Affiliations:** ^1^Department of Information Systems, Faculty of Computing and Information Technology, King Abdulaziz University, Jeddah, Saudi Arabia; ^2^Department of Civil Engineering, Mizan-Tepi University, Ethiopia

## Abstract

As online shopping has expanded, product recommendations on e-commerce websites have gained significance. Systems for recommending products use information about site navigation and user leave-over to suggest more products. Customers who use a product recommendation system choose better and find items more quickly. On e-commerce websites, collaborative and content-based filtering is used in product suggestion algorithms. Collaborative filtering is driven by user preference similarity and content-based filtering. While content-based filtering groups are related to products, collaboration groups are like-minded individuals. In collaborative filtering, users with similar user profiles are used during the proposal phase; in content-based filtering, users with similar product profiles are found and recommended. These techniques cannot deliver complex commodities and have slow start-up times and small element sets. Users can push the same product if they only like certain things, but they cannot recommend a new product or user who just joined the system because they are not a group member. These approaches cannot capture complex semantic relationships, making them inadequate for recommending complex products. Recent research has focused on incorporating the domain ontology into the proposition process to create a more precise and helpful suggestion. The relational qualities of the product are not covered in this study, only its category and features are. Actually, the ontology of the proposed product should be included in the suggestion system. Relational data is integrated into the recommendation engine in this study using domain ontologies. This was done to research books that people had recommended. Relational data from an online bookseller was used to test the proposed infrastructure.

## 1. Introduction

Electronic commerce is becoming more and more popular as a result of how simple transactions are. Still, the sheer number of products available on e-commerce websites makes it challenging for customers to find what they are looking for quickly. While browsing websites or viewing potentially interesting products, suggestion systems assist users in making decisions. [1] Recommendation systems use user data to present customers with goods that might be of interest. Both Pandora and Amazon use recommendation engines. Competition has spawned a variety of strategies to boost the success of these sites' user suggestions as a result of the rapid growth of electronic commerce websites. Systems that recommend products use CF and CBF (content-based filtering) [2].

The article "Ontology-Based Relational Product Recommendation System" was published in 2022. Journal: Comput Math Methods Med.

User preferences determine collaborative filtering (CF). Users are grouped based on features they share or like, and the group most closely matches the user profile for the suggested user is chosen. CF experiences issue with sparsity and cold starts [3]. Because no one has previously liked it, new content (product) added to the system will not be recommended to users. Users can show their preferences by visiting the page, buying the content, or casting votes. A new user without a preference cannot be recommended because CF is based on user preferences. If only a few user-favored contents exist, the same content will always be suggested [4]. In CBF, contents (products) are categorised into groups based on their unique traits. The group most closely resembles a user profile that represents the user is identified and a recommendation is made. A user's profile is created based on the content that has been bought, liked, or visited. The variety and complexity of CBF's products are both limited. Non-CBF content cannot be recommended to users [5]. Another issue is the CBF's inability to suggest complicated products. CBF is unable to record product semantics. The film's director or the course's student is ignored if a product is only represented by its attributes [6].

Hybrid studies combine the two to fix their shortcomings. Both can be combined using various techniques. The results can be weighted or some CBF features can be incorporated into the IP method. Both methods can be used independently [7].

Current research suggests more accurate products using ontologies to solve CF and CBF problems. Ontology is a conceptualization, according to Gruber [8]. Examples, relationships between concepts and ontologies are all included. Utilizing ontologies allows you to take advantage of the deep semantic qualities of objects and improves your chances of successfully proposing complex objects [9].

### 1.1. Purpose of the Work

A homogeneous structure is presumed in many studies of ontology-based product propositions. Ontologies were treated as a single class in these studies, and/or complex class attributes were disregarded.

Since these class components also influence user preferences, ontologies should include other classes to which the proposed class is related. There are two factors to consider when predicting a product's success: the product itself and the company's reputation. An additional feature of this type of data set is the possibility of a variable number of linked objects for each product and a multivalue property. In Figure 1, we see domain ontology. There will be proposed objects for Class C1. Class C1 is the “target class,” related to class C2, and has characteristics A1 and A2.

The article "Ontology-Based Relational Product Recommendation System" was published in 2022. Journal: Comput Math Methods Med.

Class C2 has its characteristics and is a subclass of class C1 as a result (A3 and A4). A book recommendation system may assign C1 to the book class, A1 and A2 book classes' subject and publication year requirements, and C2 to the author class, awards A3 and A4 authors have won, and age requirements.

This study creates a new relational, semantic, and ontology-based suggestion system infrastructure. The study starts by using coefficients to weigh the attributes of the proposed products and related products. Attribute coefficients were calculated using a CF-based method and a genetic algorithm. The proposed infrastructure is in 5 stages. First, user sessions are created from the website's access logs. Visited products are included in user sessions. Second, subclass attributes are added to the list of product attributes. Next, attributes are weighted by genetic algorithms. In the fourth stage, third-stage coefficients are used to aggregate the attributes of e-commerce websites to condense the search space. A proposal is the last step. Products from the cluster that is most near the last item the user viewed are recommended to them. A web bookstore was used to develop and test a relational and semantic suggestion model based on ontologies. Other products can use the infrastructure.

Product recommendation systems make use of ontology-based studies. Most of these studies map user-visited web pages to ontology class objects, transform the user's web page sequence into an operation sequence of ontological objects, and apply data mining methods to the resulting sequence of operations. Many studies have treated ontology as a single-class data structure, ignoring its relational structure.

An ontology-based web page is described by Dai and Mobasher [10]. The engine aggregated web page sessions into a single object after converting them to ontology objects. For each attribute, join functions are assumed. Each object has a coefficient in aggregation functions that combine session objects into one. In sessions, coefficients were used as page visits. Clustering occurs following the merge process for each session. A merge function object represented the proposed active session, and the cluster center closest to this object was determined. The proposal's implementation in the study is unclear.

## 2. Methodology

Recommended model: the model proposed in this study consists of 5 basic operations: session identification, session extension, determining coefficients, clustering, and suggesting.

The article "Ontology-Based Relational Product Recommendation System" was published in 2022. Journal: Comput Math Methods Med.

### 2.1. Session Identification

Session information can be found in cookies, proxy servers, application interaction data, or web server access logs [11]. Logs from a server's website are routinely mined for information about user sessions when more reliable sources are unavailable. Web server access logs contain information such as date, time, client IP address, browser version, accessed page URL, and request status. In web server access log analysis programmes like LogParser [12], the necessary fields are filtered to combine these records. Some access log entries are ineligible for use as session IDs. These records can be specified as

- Requests with status codes other than 200. These requests resulted in an error
- Multimedia file requests such as image files. The URL field of these requests does not correspond to a web page
- Spiders created records. Whether or not a record was created by the spider can be determined from the client browser version

The records, as mentioned earlier, which will not be used in session determination, are cleared from the access log. A page set “*P*” containing a list of all requests and a total of *m* different pages found in these requests is obtained.

(1) $$\begin{array}{c} P=\langle p_{1},p_{2},\cdots ..,p_{m}\rangle \cdots . \end{array}$$

Unique users are detected to identify sessions. Unique users are determined by assuming a user will have the same IP and client browser version. A session starts with the first request by the user and ends after a certain period of inactivity. This time is 20 minutes for most web servers. Sessions are determined from the access information and take into account individual user information and inactivity time. At the end of this stage, a session set *S* consisting of web pages is obtained. The *n*-dimensional Si session in the *S* cluster is specified in (2).

(2) $$\begin{array}{c} S_{1}=\langle p\prime_{1},p\prime_{2},\cdots ..,p\prime_{n}\rangle \text{ such that }p_{k}^{n}\in P,\text{so and }1\leq k\leq n\cdots . \end{array}$$

Each web page assumes a single product, so common pages with multiple products are ignored. In order to reflect the web pages on the ontology, the ontology of the product on the pages should be learned first.

Ontology can be learned with natural language processing techniques or an ontology with the same content that has been created and accepted before can be used. The ontology used in this study was created manually because it has been stated in previous studies that it is more convenient to create the ontology manually for small and static websites [10]. Usable information about the product on each web page in the *P* cluster is obtained with manually developed or available information extraction tools [13]. Individuals belonging to the ontology are created with this information. The available information here is the attributes of the classes in ontology. The projection of web pages to objects belonging to classes in ontology is shown in Figure 2.

The article "Ontology-Based Relational Product Recommendation System" was published in 2022. Journal: Comput Math Methods Med.

After the objects belonging to the class in the ontology are determined, the example session in (2) is converted to contain the objects belonging to the classes in the ontology to which these pages are reflected, instead of Si web pages. “*O*” is represented by the *n*-element *Si* session (3), with the set of objects of class C1.

In the proposal stage, since information about which page is reflected on which object is required, a table recording the pages and the objects they are reflected in is created at this stage.

### 2.2. Determining Coefficients

In the similarity calculations, the attributes belonging to the classes are weighted by assigning coefficients. Two different methods were used to determine the coefficients: both a CF-based and a GA-based approach. Due to the fact that the coefficients in both approaches ranged from 0.0 to 1.0, neither the distance nor the similarity could be more than 1.0. Coefficients are used to minimise the impact of less important features on similarity computations by giving them values near to zero.

#### 2.2.1. Genetic Algorithm-Based Method

One of the methods used in the weighting of the attributes is the genetic algorithm-based method. Each gene in this study is an attribute that needs to be assigned a coefficient, and since each chromosome contains as many genes as the number of attributes, it is a solution to the problem of assigning optimum values to attributes. Chromosomes are obtained by generating populations of randomly assigned genes. Random values assigned to genes range from 0.0 to 1.0. This method aims to assign a high coefficient value to the attributes that are important for the user to make a choice. An example of gene, chromosome, and population is given in Figure 3.

The fitness value of chromosomes is the ratio of the number of successful suggestions to the total number of suggestions by using the genes in the chromosome as coefficients.

In Figure 3, protect patients' privacy, it is essential to give the supplied medical images protection. Encryption and watermarking are necessary for secure transmission to maintain data integrity and confidentiality. Enhancing cryptography requires the use of encrypted data. The chromosomes undergo additional crossings, such as *j* and (*p* + 1 − *j*), which can endure various attacks for a long time. The proposed method is based on number theory and the Chinese remainder theorem. This technique delivers a high level of security and long-lasting resistance to numerous threats.

The article "Ontology-Based Relational Product Recommendation System" was published in 2022. Journal: Comput Math Methods Med.

To determine which chromosomes to cross (Selection) [14]:

- All chromosomes are ordered according to their fitness values
- *i* and (*i* + 1) Crossover is applied as long as *i* < (*P*/2) + 1 between the chromosomes. *P* is the number of chromosomes in the population
- Other crosses *j*. and (*p* + 1 − *j*) applied to the chromosomes

Thus, half of the crossovers occur with the chromosomes with the highest fitness value. The other half of the crossovers is performed between the chromosomes with the highest fitness value and those with the lowest fitness value. In these crosses, since the fitness value of one parent is higher than the other, the fitness value of the next generation chromosome is expected to be higher than that of at least one parent.

The crossovers were performed not in the form of gene exchange in classical genetic algorithms but combined with some kind of mutation by taking the arithmetic average of the parents. The arithmetic mean of the genes in the parents is assigned to the son genes in the same order. Thus, the genes in the new generation chromosomes are formed between 0.0 and 1.0. The crossover ratio was taken as 1.0 and all chromosomes were crossed over. The flowchart of the method of determining the coefficients by crossing an *n*-dimensional population by *K* is given in Figure 4 and an example of crossover and mutation are given in Figure 5.

### 2.3. Session Extension

In Section 2.1, sessions are obtained to consist of objects of the class in ontology. Some of the attributes of this class may also be a class with its own attributes. We will call such classes' subclasses. Subclasses have their own attributes and are attributes of another class. In the sessions obtained in Section 2.1, these subclasses are represented only as an attribute with names. In the session extension phase, the domain ontology and ontological objects belonging to these subclasses are created and the sessions are extended to include both the target class object and the subclass object. At this stage, the ontology was created manually and the objects belonging to the class in ontology were obtained with information extraction tools as indicated in Figure 3. The sample session Si formed at the end of this stage is given in (4). ‘SO' is the set of objects belonging to the C2 class specified in Figure 5. The main point here is that the session given in (3) consists of objects belonging to class C1 only, while the session given in (4) consists of both objects belonging to class C1 and objects belonging to class C2. In a real dataset, class C1 may oppose the book class and class C2 may oppose the author class. For sessions consisting of this dataset, (3) only has objects of the book class, while (4) has objects of both the book class and the author class. While in (3) the author is only a noun, in (4) it is a subclass with its own characteristics (age, awards, etc.).

The article "Ontology-Based Relational Product Recommendation System" was published in 2022. Journal: Comput Math Methods Med.

In this study, the number of crossovers was repeated at a predetermined number (*K*), but the crossover could be repeated until a fitness threshold value was reached. Results were produced for different values of *N* (number of chromosomes in the population). As a result, the genes in the chromosome with the highest fitness value were taken as the coefficients of the attributes.

#### 2.3.1. Collaborative Filtering-Based Method

Users' navigation on electronic commerce websites varies with the characteristics of the product class [15]. For example, for a site that trades books, some users browse only by paying attention to the subject of the book, or because some users may only be interested in new books, they only visit the pages on the site with the content of new books. The purpose of the CF-based method is to find out for which attributes users prefer a product and to identify these attributes as important attributes and others as unimportant ones.

After the insignificant features are determined, a coefficient lower than 1.0 is assigned to these features, reducing their effect in the similarity calculation; coefficients are not assigned to important attributes, leaving 1.0. To identify important and unimportant attributes

- A vector is generated for each attribute of the objects in the sessions
- A purity function is used to find the purity in vectors. Purity is the determination of how different or how similar the elements in the vector are. If all the elements in the vector are the same, the purity is maximum; if they are all different, then purity is minimal. The purity function used in this study compares all the elements in the vector with each other and takes the ratio of the number of element pairs determined to be the same as a result of these comparisons to the total number of comparisons as the purity value
- A session set of randomly generated sessions is obtained. The content of these sessions is randomly selected from the members of the sessions in the session set obtained in Section 2.1. The sizes of the sessions in this randomly generated session set are the same as the sizes of the sessions in the session set obtained in Section 2.1. For example, if there are a total of *N* sessions of size *K* in Section 2.1, *N* sessions of size *K* will also be created in the randomly generated session set. Thus, two different session sets are obtained; the session set obtained from the web server access log in Section 2.1 and the randomly generated session set
- For each attribute of the classes in the ontology, the average purity value (APV) of the sessions in both the session set obtained from the access log and the randomly generated session set is calculated. The coefficient of the attributes in the class is determined using the APVs as shown in

(3) Ratio=XY X=APV of sessions generated from access log files. Y=APV of randomly generated sessions K=A predetermined threshold value. Coefficient=1If ratio>K=Maximum Ratio,0.9If ratio<K

How much an attribute affects the user's preference is determined by the ratio value in (2.9). If it is less than the threshold value, this attribute is considered unimportant, and the ratio value is determined as the coefficient is taken. If this value is between 0.9 and the threshold value (*K*), the coefficient will be taken as 0.9.

The article "Ontology-Based Relational Product Recommendation System" was published in 2022. Journal: Comput Math Methods Med.

### 2.4. Clustering and Similarity Calculations

The normalized database system is very similar to the structure produced in Section 2.2. A relational database schema is an ontology [10] because it comprises numerous tables linked semantically and through foreign keys. Therefore, relational database methods are suitable for the structure obtained in Section 2.2.

The first problem of this structure is to determine how to handle subclasses and their attributes when measuring similarity or distance. In this study, 2 different similarity calculations using cosine similarity and 3 different Euclidean distance calculations were implemented.

First cosine similarity (CS) was computed using only target-class attributes as input. Both the target class and the subclass properties were used in the second cosine similarity computation. For example, in the calculation of book similarity, the attributes of the author class were also taken as input. This calculation is called “Extended Cosine Similarity” (ECS).

The only ones used in the first Euclidean distance (ED) computation were attributes unique to the target class. Attributes of the subclass were also used as input in the second and third Euclidean distance calculations. For this reason, objects belonging to the subclass are obtained in Section 2.2. The difference of the second and third Euclidean distance calculations of the second; the third is to calculate the distance. The second calculation in this study is “Extended Euclidean Distance-1” (EED-1); the third calculation is called “Extended Euclidean Distance-2” (EED-2). Since all attributes are normalized, distance values vary between 0.0 and 1.0. So the distance between O_1_ and O_2_ objects can convert to similarity as follows:

(4) $$\begin{array}{c} \text{Similarity }\left(O_{1},O_{2}\right)=1-\text{Distance}\left(O_{1},O_{2}\right). \end{array}$$

Another problem in relational structures is multivalued attributes. Some attributes of classes can be multivalued. For example, a movie has more than one actor. Generally, concatenation functions that reduce multivalued attributes to a single value are used to solve this problem [16]. The CS, ECS (extended cosine similarity), SS, GS-1, and GS-2 methods used in this study have been developed to work on multivalued attributes. These methods consider the similarity between the multivalued attributes of two objects as the ratio of the number of elements at the intersection of the respective attribute value sets of the objects to the number of elements in their union. For O_1_ and O_2_ objects, *f* (O_1_), and the number of elements belonging to the value set of a multivalued attribute of the O_1_ object, the similarity of the related attributes of these objects is calculated. The similarity calculation for numeric multivalued attributes is achieved by finding the similarity of each value in the value set of the O_1_ object with each value in the value set of the O_2_ object and calculating the arithmetic mean of these. Since the similarity calculation method is adapted to calculate multivalued features, traditional distance-based clustering techniques such as *K*-means can be used on data. It is aimed to narrow the search space with clustering. In the similarity calculations at the clustering stage, the attributes were weighted by assigning coefficients. The determination of the coefficients is explained in Section 2.3.

The article "Ontology-Based Relational Product Recommendation System" was published in 2022. Journal: Comput Math Methods Med.

### 2.5. Making Suggestions

At the suggestion stage, the last visited page by the active user is taken into account and the object of this page reflected in the domain ontology is determined. In the next step, the nearest cluster center is determined by calculating the distance of this object to the cluster centers and the distance to the objects in the nearest cluster are calculated. The web pages corresponding to the *N* objects in the cluster closest to the object in the active session are presented to the user as suggestions. Which web page is reflected on which object is determined and recorded in Section 2.1. These processes are visualized in Figure 6.

## 3. Results

### 3.1. Implementation of the Product Recommendation System

The website's ontology for the product (book) was created manually. There are two classes in the created book ontology: book and author. Publisher class is not included in the ontology since the publisher is the same for all books. The book class is the target class whose objects will be suggested. On the other hand, the author class is a subclass because it is both a class with its own attributes and an attribute of the target class. The characteristics of the book class specified as follows:

- Area: a double-precision floating-point number type attribute that represents the book's physical dimensions; corresponds to the product of the width and height of the book
- Publication Year: it is an integer type attribute that indicates the last publication year of the book
- Binding Type: a Boolean attribute that indicates whether the book is bound or paperback
- Price: a double-precision floating-point number type attribute specifies the book's price
- Quality: a double-precision floating-point number type attribute that specifies the book's paper quality, 1.00 for coated paper; 0.66 for 1st pulp paper. It is accepted as 0.33 for the 2nd pulp paper and as 0.00 for the 3rd pulp paper
- Category: it is a string-type attribute that specifies the book's subject.
- Author: it is a class variable that specifies the book's author
- New Publication: a Boolean data type attribute indicates whether the book was published in 2020 or not

The attributes of the author class are specified and explained below:

- Date of Birth: an integer type attribute that specifies the date of birth of the author. To avoid outliers, the minimum value of 1900 was accepted, and the value of this attribute was taken as 1900 for authors with a birth date before 1900
- Number of Books: it is an integer type variable that indicates the number of books published by the author from Yapı Kredi Publications
- Categories: it is a string type variable that consists of the categories of the books written by the author before

After defining the domain ontology, the website's products are added. These products' web page information was extracted using software. Information extraction tools are implemented in C# to display the web page's source code and extract necessary information using regular expressions. Regular expressions have been the best method for years [17, 18]. Product information was obtained by defining a repeating regular expression in the web pages' source code.

First, the Yapı Kredi Publications website was searched for author and book class information. We have tried to get information from Kibo's website. The missing information was gathered from other sources. 2222 books and 925 authors' objects were defined.

CS, ECS, ED (Euclidean distance), DS-1, and DS-2 were used to determine the distances between the defined book objects.  Section 3.3.1 contains test results and clustering details.  Section 3.3.2 explains the successful coefficient assignment methods.

The article "Ontology-Based Relational Product Recommendation System" was published in 2022. Journal: Comput Math Methods Med.

Calculating coefficients uses ontology-based sessions. The LogParser programme combined web server access log files and removed extraneous records to identify sessions. The session did not include a multiproduct page. IP address and client browser version were used to detect single users, and 20 minutes of inactivity was used to identify sessions. Only more than one size sessions were considered to evaluate the proposed system's effectiveness. The 55-day logs contained 4317 sessions, 2791 of which were repeated. Multiple-size sessions average 3.18. Sessions begin with web pages because the objects on them are preobtained. Sessions consist of the products on these pages, not web pages. Sessions were created using book class objects. Next, book and author class objects are added to the sessions.

### 3.2. Evaluation Criteria

The proportion of implemented suggestions as a percentage of total suggestions was accepted as the metric necessary to assess the effectiveness of the system. Success was defined as the discovery of the suggested product during the session, so suggestions were implemented with this in mind.

### 3.3. Performance Tests

#### 3.3.1. Similarity Calculation Methods Tests

The success results of the ontology-based relational product recommendation system were compared with the success results of an alternative approach using the Markov chain model. This model was chosen for comparison because it has been demonstrated in numerous studies [19] that it is successful in recommending products. The Markov chain model is a recommendation algorithm based on the similarity of user movements recorded in web server access logs. First-order and second-order Markov chain models were applied in this study. In the first-order Markov chain model, the last product visited determines the product the user will visit in the following step: in the second-order Markov chain model, it determines the last two visited products. A product's likelihood of being visited after purchase is calculated using data from the web server access log. The rates at which users can switch to a product's web page after viewing the O_1_ product's web page, for instance, are shown in Figure 7. In this instance, Ox is suggested if only one product should be recommended to the user visiting the O_1_ product.

The Markov model performance was achieved with a 10-fold cross-validation model. The 2790 sessions obtained in Section 3.1 are divided into 10 session clusters, each containing 279 sessions. Each time, 9 sets of learning sets and 1 set of test sets were used, and 10 different tests were carried out. The average success of the 10 tests according to the recommended number of books is given in Table 1. The standard deviation of the success results of the tests is 2.34 in the 1 book recommendation test and 3.12 in the 3-book recommendation test.

The article "Ontology-Based Relational Product Recommendation System" was published in 2022. Journal: Comput Math Methods Med.

The performance of the second-order Markov model was also tested with the 10-fold cross-validation model. 1240 sessions with a size of more than 2 were divided into 10 different clusters, each containing 124 sessions, and 10 different tests were performed by taking 9 learning clusters and 1 test cluster. The success results of the tests are given in Table 1. The standard deviation of the success results of the tests is 2.91 for 1 book recommendation and 4.02 for 3 book recommendation.

Second-order Markov chain models are 15% less successful than first-order models. High-order Markov models exponentially increase state space and require a large data set, leading to poor recommendation performance [20]. High-order Markov model is not good for fast web page recommendations.

Section 2.4 describes the ontology-based relational product recommendation system's CS, OA, GA, PP-1, and PP-2 methods. ECS is a cosine similarity method that uses target and subclass attributes. EED-1 and EED-2 are Euclidean distance-based methods that accept target and subclass attributes. CS and AU only use book class attributes (author, price, publication year, category, new edition, and field). ECS, EED-1, and DSS-2 used book and author characteristics (age, number of books, and book topics).

The author class's multivalued categories attribute similarity was calculated according to (4.10). The categorical similarity of the book class is 1.0 for the same category, 0.5 for the same category group, and 0.0 for different category groups. In CS and ED similarity, the author attribute is a character string, and similarity is 1.0 for the same authors and 0.0 for different authors. ECS, EED-1, and EED-2 have class author attributes.

The ED, DS-1, and SS-2 methods were compared using CS and OA. Since the first test only compared the success of these methods, similarity coefficients and clustering were not performed. The most similar books to the first book in the session were suggested. In this test, a learning set of sessions or books is not needed because similarity coefficients are not weighted. Methods were tested for all sessions (2791). Figure 7 shows tests without clustering and attribute weighting.

As seen in the test results, including the characteristics of the subclass in the similarity calculation increased the success. For example, CS's success in the 3 book recommendation test was 17% when it only used the attributes of the book class, while it was 26% when it used the attributes of both the book and the author class. The success rate in the AU method is 34%, increasing to 44%. There are 2.4 books per author in the dataset. For this reason, since only the name of the author cannot be a good distinguishing feature for books, using the attributes of the author class has increased the success.

The article "Ontology-Based Relational Product Recommendation System" was published in 2022. Journal: Comput Math Methods Med.

In the second test, the books were clustered and after the closest cluster to the first object in the session was determined, the closest objects in this cluster were suggested. Since similarity calculations are performed with the extended forms of traditional methods (cosine similarity and Euclidean distance) to operate on relational data, no tool was used for similarity calculation. Similarity calculations were made with a programme implemented in C# and a similarity matrix was created. Clustering is implemented with the cluster bundling method in the CLUTO software tool [21], which accepts the similarity matrix of the objects to be clustered as input. Clustering was carried out using the stacked hierarchical method with the “agglo” key of the cluster method.

The stacked hierarchical clustering method consists of the following steps:

- Each object is considered as a separate set, denoted by *G*1, *G*2, ⋯, *Gn*, and the similarity matrix of these objects is calculated
- Number of n clusters in the similarity matrix, *i* = 1, 2, ⋯, *n*, *j* = 1, 2, ⋯, *n*, and *i* ≠ *j*

Two clusters with at least *D* (G_i_ and Gj) distance are determined and a new cluster is formed by combining these two clusters.

- The similarity matrix is updated considering the newly formed clusters
- The above steps are repeated until a single cluster is obtained (until the root of the dendrogram is reached)

The achievement test results for the case where the number of clusters is 5 are given in Figure 8. Achievement test results for the case where it is 10 are given in Figure 9. Since the qualifications were not weighted in these tests, there was no need for a learning set, and the tests were performed on all sessions.

After the books are clustered first, the closest cluster is determined. In the case where the closest books are recommended, for 5 clusters, success decreased by about 28%, search space shrunk by 63%. For 10 clusters, the success decreased by about 40% and the search space was reduced by 71%.

Similarity calculations can be performed offline based on sessions' last visited web page. In this case, narrowing the search space may not be important, but when the last *N* products in the sessions are reduced to a single product with the aggregation function, online similarity calculations will be more important. Clustering the products can narrow the search space because the decrease in success rate is less than the shrinkage rate of the search space. Since the test data set's search space is small, clustering was not performed in 3.3.2's feature weighting tests.

The article "Ontology-Based Relational Product Recommendation System" was published in 2022. Journal: Comput Math Methods Med.

#### 3.3.2. Attribute Weighting Tests

GA and CF weighted attributes differently. In weighting attributes with GA, a population of 11 genes (7 for book class attributes and 4 for author class attributes) was created. Crossovers and mutations increase the fitness of the population's chromosomes. Fitness value is the recommendation success rate based on chromosome genes.

The CF-based method creates a random session set with the same dimensions as the web server access log. 1542 sessions with a size of 2 are randomly generated in the newly created session set when we obtain the sessions from the web server access log as explained in Section 2.1. Randomly created sessions are made from access log sessions. Section 2.3's APV was calculated for both session sets (obtained randomly from the access log). *K* in (4.9) was experimentally determined as 1.20 when determining attribute coefficients. An attribute is considered important if it affects the user's product choice by 20%.  Table 2 shows success rates by *K* value (threshold). Both methods were cross-validated 10 times. 2790 sessions were divided into 10 session sets, including 279 sessions. Nine session sets were used as learning sets, and 1 session set was used to test the coefficients.  Table 3 shows the GS-1 weighting test results. Success ranges from 44% with CI to 62% with CF. Success was increased by removing unimportant user preferences from the similarity calculation. In GA, the standard deviation of test success is 1.08 for the 1-book and 1.39 for the 3-book tests; in CF, it is 1.37 for the 1-book and 3.87 for the 3-book tests. In GA, the variance of test success is 1.16 for 1 book and 1.93 for 3 books; in CF, it is 1.87 for 1 book and 14.97 for 3 books.

The Mann–Whitney *U* test can determine the statistical significance of two groups whose elements are not matched and do not show normal distribution [22]. For this reason, the Mann–Whitney *U* test was used to determine the statistical significance of the success of the proposed model compared to the success of the Markov chain model. It has been determined that the success of the proposed system, in which the GAU-1 method and the GA method are used, shows a significant difference at *p* < 0.005 significance level compared to the success of the Markov chain model and significantly increases the success. (*p* = 0.0002).

The article "Ontology-Based Relational Product Recommendation System" was published in 2022. Journal: Comput Math Methods Med.

The crossover ratio was taken as 1.0 in the weighting of the features with GA, and all chromosomes were crossed and obtain the next generation chromosomes. Different success rates have been obtained using various population sizes and various crossover repetitions. The effect of the number of crosses and the number of chromosomes in the population on success is given in Figure 9.

The second GS-1 test recommended a product based on the user's last two visits. This test suggested products at the intersection of the user's last and penultimate visits. If the number of products at the cluster intersection is less than the number to recommend, the last visited product's recommendation set suggests similar products.

The success of this test was realized by using a 10-fold cross validation model by dividing 1240 sessions with a size larger than 2 into 10 clusters. Test results are given in Table 4. In the achievement test of the CF-based method, the standard deviation was 2.09 in the 1 book recommendation and 4.77 in the 3-book recommendation. In the achievement test of the GA-based method, the standard deviation is 1.75 for 1 book recommendation and 2.43 for 3 book recommendation. It has been determined by Mann–Whitney *U* test that the success of the proposed system according to the last two products is significant at the *p* < 0.005 significance level compared to the success of the second-order Markov chain model and significantly increases the success. (*p* = 0.003).

In the case of assigning coefficients to the attributes in the ECS method, the similarity calculation formula specified in (2.14) is *W*^*i*^ and *i*. The coefficient of the attribute will be as follows:

(5) $$\begin{array}{c} S\left(O_{1},O_{2}\right)=\frac{\sum_{i=1}^{n}O_{1}^{i}\times O_{2}^{i}W^{i}}{\sqrt{\sum_{i=1}^{n}{\left(O_{1}^{i}\right)}^{5}}+\sqrt{\sum_{i=1}^{n}{\left(O_{2}^{i}\right)}^{5}}}. \end{array}$$

Similar to the GU-1 method, a 10-fold cross-validation test was used with the ECS method. In the GA test, the population's 25 chromosomes were assumed, and crossover was applied 100 times.  Table 5 provides the ten test results' average success rates. The tests' standard deviations in CF were 1.09 for a single book recommendation and 1.16 for three; in GA, the values were 0.67 for a single book recommendation and 1.34 for three. In CF, the variance of the tests was 1.18 for a single book recommendation and 1.34 for three, whereas in GA, it was 0.44 for a single book recommendation and 1.79 for three. As in the PP-1 method, reducing their effects by giving low coefficients to insignificant attributes in the ECS method increased the success of product recommendation. The proposed system, which combined ECS and GA techniques, was found to perform significantly better than the Markov chain model at the 0.05 significance level, according to the Mann–Whitney *U* test. (*p* = 0.01 and *u* = 15.5).

The article "Ontology-Based Relational Product Recommendation System" was published in 2022. Journal: Comput Math Methods Med.

## 4. Conclusion and Recommendations

Deep semantic relationships between products are used in ontology-based product recommendation systems to increase performance and address issues like cold start, element sparsity, and limited diversity in CF and CBF methods, which are frequently used in product recommendation systems. The concepts in a specific field and their relationships are the fundamental components of ontology. As a result, the product's class and any other classes, it has relationships with must both be included in the ontology of the product. This kind of structure is a relational data structure, and ontologies can be mined for data using relational data mining techniques. From this perspective, a relational product recommendation system that makes use of domain ontologies has been developed, tested, and proven to be very effective. According to experimental findings, including additional classes that the product is related to increases its success. The study also highlights the need to weight the attributes by allocating coefficients. Not all characteristics of a product stand out to users. The success has increased by identifying the attributes that do not influence users' preferences and minimising the effects of the similarity calculation by keeping the coefficients of these attributes low. The proposed system has been tested using experimental findings for book ontology, but it can also be used with ontologies for other kinds of products. Future work is encouraged on intriguing issues like defining a join function that can represent an ongoing session with an object of a class in the domain ontology.

## Figures and Tables

**Figure 1:** Abstract domain ontology.

**Figure 2:** Projecting web pages to ontology individuals.

**Figure 3:** Protecting web pages for ontology medical image with security applications.

**Figure 4:** Flowchart of coefficient determination with GA (Genetic Algorithm).

**Figure 5:** Crossover and mutation.

**Figure 6:** First-order Markov chain.

**Figure 7:** Similarity calculation methods performance rates.

**Figure 8:** Similarity calculation methods performance rates for 5 clusters and for 10 clusters

**Figure 9:** Chromosome count and crossover repeat count in the population.

**Table 1:** First- and second-order Markov chain success rate.

Recommended number of books	First-order Markov chain success rate	Second-order Markov chain success rate
1	14.50%	12%
3	36%	32%

The article "Ontology-Based Relational Product Recommendation System" was published in 2022. Journal: Comput Math Methods Med.

**Table 2:** CF-based attribute weighting achievements according to *K* value.

*K* value	Success rate
1.1	49%
1.2	58%
1.3	51%
1.4	50%

**Table 3:** Achievements of attribute weighting methods in GS-1 method.

Number of books recommended	Methods			
	First-order Markov chain	Without weighting	CF based	GA
1	14.50%	17%	25%	27%
3	36%	44%	58%	62%

**Table 4:** Achievements of GS-1 and attribute weighting methods -2.

Number of books recommended	Methods			
	Second-order Markov chain	Without weighting	CF based	GA
1	12.30%	16%	22%	23%
3	31.80%	42%	52%	55%

**Table 5:** Achievements of attribute weighting methods in ECS method.

Suggested	Methods		
Number of books	Without weighting	CF based	GA
1	0.07	0.15	0.17
3	0.17	0.35	0.39

## Data Availability

The data underlying the results presented in the study are available within the manuscript.
